The article "An Empirical Study on Physical Subhealth Risk Perception: A Physical Examination Data of Tertiary Grade-A Hospitals in Anhui Province, China" was published in 2023. Journal: J Environ Public Health.

# An Empirical Study on Physical Subhealth Risk Perception: A Physical Examination Data of Tertiary Grade-A Hospitals in Anhui Province, China

**DOI:** 10.1155/2023/3959571

**Published:** 2023-01-30

**Authors:** Xueli Jiang, Liping Zhang, Yufei Gao, Chengsen He, Zhiru Tang, Jiangjie Sun

**Affiliations:** ^1^School of Health Care Management, Anhui Medical University, Hefei 230032, China; ^2^School of Marxism, Anhui Medical University, Hefei 230032, Anhui, China; ^3^Law School, Anhui Medical University, Hefei 230601, China

## Abstract

**Background:**

Physical subhealth directly correlates to people's work effectiveness and quality of life, so subhealth prevention has become an urgent medical problem.

**Methods:**

A random sampling method was used to conduct a questionnaire survey of physical examinees from June to September, 2019. In total, 770 people participated in our study. The Pearson correlation and multiple stepwise regression analysis were used to explore the relationship among demographic variables, physical subhealth, and risk perception. Also, this study used a two-way interaction moderated multiple regression approach to examine the moderating effects of demographic variables on physical subhealth and risk perception.

**Results:**

The risk perception level was negatively associated with physical health. Age, education level, and subhealth proportion in the work unit all significantly and positively influence physical health, whereas living place, subhealth duration, and marital status negatively influence physical health. Living place, average annual household income, number of employees in the work unit, and subhealth proportion in the work unit significantly and positively influence the risk perception, and only age negatively influences the risk perception. The number of children had a moderating effect on physical subhealth and risk perception (Interaction coefficient *α* = −0.3, *P* < 0.05).

**Conclusions:**

To achieve the overall improvement of public health, relevant management departments can provide targeted interventions for the public with different levels of risk perception. Also, the physical subhealth of the public can be addressed by encouraging the public to attach importance to education, improving the public living environment to build a livable city, strengthening psychological guidance and intervention for couples heading toward divorce to reduce the divorce rate, focusing on the health of work unit employees and regularly organizing employees to attend medical checkups, and actively responding to the national policy of family planning.

## 1. Introduction

In 2006, the Clinical Guidelines of Chinese Medicine on subhealth, issued by the China Association of Chinese Medicine [1], pointed out that subhealth refers to a state of human body between unhealthy and healthy. A subhealthy person shows symptoms of decreased vitality, function, and adaptability within a certain period but does not meet the clinical or subclinical diagnostic criteria of modern medicine's defined diseases. This condition is also known as a “grey state” or “third state.” Subhealth includes symptoms such as physical fatigue, psychological anxiety, depression, and decline of social adaptability, which seriously affect people's quality of life. The process of body life is the mutual transformation of health, subhealth, and disease. Without timely intervention, subhealth will lead to the occurrence of diseases [2]. A study pointed that only 5% of the global population were in a complete health state, 20% were in a disease state, and the remaining 75% were in subhealth status [3]. Individual physical subhealth is a global public health problem that needs to be solved urgently.

The article "An Empirical Study on Physical Subhealth Risk Perception: A Physical Examination Data of Tertiary Grade-A Hospitals in Anhui Province, China" was published in 2023. Journal: J Environ Public Health.

### 1.1. The Relationship between Physical Subhealth and Risk Perception

Risk perception, which reflects people's cognition and intuitive judgment of risk [4], is studied in the field of psychology [5]. Risk perception is one of the core elements of health behavior theories; those theories point out that people exposed to risk are motivated to stop unhealthy behaviors and adopt healthy behaviors to avoid negative consequences [6]. For example, the health belief model [7, 8] takes susceptibility and severity to disease as pretest factors of whether an individual adopts healthy behaviors, where the cognition of susceptibility to disease and severity is the risk perception. The protective motivation theory [9, 10] explains why health behaviors occur from the perspective of motivation, in which risk perception plays a central role. The level of risk perception affects the behavioral lifestyle of the public [11], while lifestyle is one of the most important factors influencing health status. Positive risk perception attitudes of the public play a key role in driving individual adaptive behavior and are a precondition for the public to make healthier lifestyle choices, participate in health screenings, and adhere to health care [12]. People with higher risk perception levels are more likely to resist unhealthy behaviors and adopt healthy lifestyle habits, which helps to increase their level of self-protection against risks and reduce health threats due to various risks [13, 14].

### 1.2. Current Study

Domestic and international scholars have carried out numerous studies on subhealth, but those research efforts mainly focused on the diagnosis [2], influencing factors [15], and treatment options [16] of subhealth, while there was a relative lack of research on the prevention of subhealth. Many studies exploring risk perception have pointed out that demographic variables are significantly related to risk perception and risk reduction behaviors. For example, relevant studies showed that risk behavior decreases with the increase of age [17], the level of risk perception in women was higher than that in men [18], education level was negatively correlated with risk perception level [19], and higher income will reduce the occurrence of risk behavior [20].

The article "An Empirical Study on Physical Subhealth Risk Perception: A Physical Examination Data of Tertiary Grade-A Hospitals in Anhui Province, China" was published in 2023. Journal: J Environ Public Health.

This study explores the influencing factors of physical subhealth from a new perspective of risk perception, analyzes the mechanism of action between risk perception and physical subhealth, and discusses the moderating effects of demographic variables and related control variables on physical subhealth and risk perception. This work provides a theoretical basis for reducing public subhealth risk and provides a judgment basis for health warnings. Thus, based on the previous research, we propose the following hypothesis.

**Hypothesis 1 .**

Risk perception level positively influences physical health.

**Hypothesis 2 .**

Physical subhealth negatively influences individual risk perception.

**Hypothesis 3 .**

Many demographic variables and control variables impact the level of risk perception.

**Hypothesis 4 .**

Many demographic variables and control variables impact physical subhealth.

The conceptual model is shown in Figure 1.

## 2. Methods

### 2.1. Study Design and Study Population

This was a cross-sectional study performed in four grade-A hospital physical examination centers in Anhui Province to obtain data on physical subhealth and risk perceptions of physical examinees. The study period was from June to September, 2019. Anhui's economy has been developing rapidly in recent years, and its comprehensive strength has been steadily improved. With the booming economy, the pressure on people in all areas is also increasing, and the public's health status has attracted much attention. This study selected examinees at physical examination centers as the research participants and explored the relationship between the public risk perception level and physical subhealth status. Participants were excluded if they did not give verbal consent prior to the start of the questionnaire or refused to cooperate with this study while the questionnaire was in progress. Participants who gave verbal consent to participate in this study before questionnaires were selected, thereby ensuring that participants were voluntarily agreeing to participate in the study. In this study, a total of 785 questionnaires were collected from physical examinees by our random sampling method, and 770 valid questionnaires were obtained after excluding invalid questionnaires, yielding a response rate of 98%.

The article "An Empirical Study on Physical Subhealth Risk Perception: A Physical Examination Data of Tertiary Grade-A Hospitals in Anhui Province, China" was published in 2023. Journal: J Environ Public Health.

### 2.2. Ethical Approval and Consent

Our study was approved by the Ethics Committee of Anhui Medical University (No. 20190463). Human rights and ethics issues were taken into consideration when the survey was designed. To save participants' time, verbal informed consent was obtained from each participant following a detailed explanation about the purpose of the study. For participants under the age of 18, verbal informed consent was obtained from their parents or legal guardians. Participation in the study was voluntary and anonymous, and the participants' information was kept completely confidential. All procedures performed in studies involving human participants were in accordance with the Declaration of Helsinki.

### 2.3. Measures Used

The survey was administered by researchers assisted by undergraduate students majoring in health management, master of health management students, professional lecturers, and associate professors. This research team was trained before distributing the questionnaires. We collected the data through the following three tools:

#### 2.3.1. Physical Subhealth Risk Perception Scale

The physical subhealth risk perception scale developed by Sun et al. was used to measure the public's perception level of physical subhealth risk [21]. The scale contained 18 items, which are divided into five dimensions. The Cronbach's*α* coefficient of the full scale was 0.889 and the Cronbach'*α* coefficients of the five factors (health knowledge, trust selection, information channel, risk perception, and social groups) were 0.704, 0.825, 0.801, 0.780, and 0.736, respectively. Structural equation model analysis showed that *χ*^2^/df = 3.43, *P* < 0.001. RMSEA = 0.08, GFI = 0.88, NFI = 0.84, AGFI = 0.84, and CFI = 0.88.

The first two items cover the dimension of health knowledge: “I am more knowledgeable about subhealth than the people around me” and “I regularly browse and read health newsletters, exam-related websites, and subhealth-related brochures.” Four items cover trust selection, asking about trustworthy agents: doctors at local community hospitals; doctors in provincial and municipal hospitals; provincial or national public health administrators; and experts/scholars at medical research institutions. Four more items concern information channels: “I obtain subhealth-related information through an Internet search (Baidu and Soso);” “I obtain subhealth related information through related hospital websites;” “I need to search for more information about subhealth;” and “I will compare this information with other relevant information.” Five items cover risk perception: total presence of subhealth indicators in an individual's body; subhealthy physical symptoms that I fear are a threat to my quality of life; subhealthy symptoms in my body and I feel anxious and scared; “Do you think the occurrence of subhealth is related to the individual's behavioral habits?;” and “Do you think the occurrence of subhealth is related to the degree of integrity of an individual's family structure?.” The social groups' dimension concerns the final three items: family members; social networks (QQ, WeChat, and Weibo); and friends, relatives, neighbors, and colleagues. Using Likert's 5-grade scoring standard, each item has five options, namely, “totally disagree,” “basically disagree,” “neither agree nor disagree,” “basically agree,” and “fully agree,” which scored 1–5 points, respectively. The total score of this five-dimensional scale ranged from 18 to 90. The higher the score, the better the individual's competence of physical subhealth risk perception.

The article "An Empirical Study on Physical Subhealth Risk Perception: A Physical Examination Data of Tertiary Grade-A Hospitals in Anhui Province, China" was published in 2023. Journal: J Environ Public Health.

#### 2.3.2. Questionnaire on Demographic Variables

The questionnaire included parts for gathering demographic data about the participants (gender, age, education level, years of working, living place, marital status, number of children, and average annual household income) and control variables data (self-assessment of health, subhealth duration, number of employees in the work unit, and subhealth proportion in the work unit). The variables are formatted as shown in Table 1.

#### 2.3.3. Self-Assessment Questionnaire for Clinical Manifestations of Physical Subhealth/Health

Based on the description of the clinical manifestations in terms of physiological functions in the Clinical Guidelines of Chinese Medicine on subhealth issued by China Association of Chinese Medicine in 2006 [22], we compiled a questionnaire to collect individual subhealth clinical data. Specifically, participants were asked if they had the following clinical symptoms that lasted for three months or longer. The clinical symptoms covered in the questionnaire include short-term knee pain symptoms; gastrointestinal and liver abnormalities (e.g., nausea in the morning, palpitations, hunger, and similar symptoms); cardiac abnormalities (e.g., shortness of breath, arrhythmia, snoring, sexual dysfunction, and similar symptoms); stool abnormalities (e.g., alternating diarrhea and constipation and long-term chronic diarrhea); and painless abnormalities (e.g., painless neck mass, painless hematuria, and similar symptoms). For each item, clinical manifestation options are divided into three categories “No,” “Yes,” and “No idea,” which scored 1, −1, and 0 points, respectively. The score of this questionnaire ranged from −5 to 5. The closer the score is to 5, the healthier the individual's body. The closer the score is to −5, the more severe the subhealth condition is.

The article "An Empirical Study on Physical Subhealth Risk Perception: A Physical Examination Data of Tertiary Grade-A Hospitals in Anhui Province, China" was published in 2023. Journal: J Environ Public Health.

### 2.4. Statistical Analysis

EpiData 3.1 software was used to establish the database and double input data. Descriptive statistics, including frequencies, percentages, means, and standard deviations, were calculated on the participants' demographic data using SPSS 23.0. Heatmap analysis of physical subhealth and risk perception data was performed using Python-3.8.6. The Pearson correlation coefficients were used to analyze the correlation among physical subhealth, risk perception, demographic variables, and related control variables. Factor analysis was used to test for multicollinearity, and multiple linear stepwise regression analysis was used to explore the effects of demographic variables and control variables on physical subhealth and risk perception. Two-way interactions in moderated multiple regression were used to test the moderating effect of demographic variables and control variables on physical subhealth and risk perception. Differences are considered to be statistically significant when *P* < 0.05.

## 3. Results

### 3.1. Demographic Characteristics of Participants

A total of 770 participants were included in the present study (male : female = 312 : 458). Among the participants, 49.9% were aged less than 30, 33.2% aged 30–45, 12.5% aged 46–60, and 4.4% aged more than 60. The average age of the participants was 34 (SD = 11.68). The average score for the self-assessment of health was −0.64 (SD = 0.88). The characteristics of other demographic variables and control variables are shown in Table 2.

### 3.2. The Effect of Risk Perception Level on Physical Subhealth/Health

In this study, two variables, physical subhealth risk perception level and clinical manifestations of physical subhealth, were used to collect data from physical examinees through a cross-sectional survey. Python-3.8.6 software was used to analyze the data of physical subhealth status and risk perception level. We found that a few physical examinees had a poor risk perception level, but most of them had a good risk perception level. As the risk perception level increased, the rate of physical subhealth status tended to increase and then decrease, peaking at the “good” risk perception level (except when the physical subhealth score was 2, which peaked at the “general” risk perception level). The details are shown in Figure 2. The results suggested that there was an effect of the public's risk perception level on physical health status.

The article "An Empirical Study on Physical Subhealth Risk Perception: A Physical Examination Data of Tertiary Grade-A Hospitals in Anhui Province, China" was published in 2023. Journal: J Environ Public Health.

*Note.* 5, 4, 3, 2, 1, 0, −1, −2, −3, −4, and −5 represent the physical health scores of the physical examinees. The closer the score is to 5, the lower the risk of subhealth and the better the health status. The closer the score is to −5, the higher the subhealth risk and the worse the health status. The risk perception score is divided into four levels according to the quartiles method [23]: 18–35, 36–53, 54–71, and 72–90. We use “poor,” “general,” “good,” and “excellent” to represent the risk perception levels. “Poor” indicates the score on the risk perception scale is 18–35, with “general” indicating 36–53, “good” indicating 54–71, and “excellent” indicating 72–90.

### 3.3. Correlations among the Study Variables

Based on the clinical manifestations and risk perception sample data for physical subhealth, Pearson's correlations were calculated among the study variables, as shown in Figure 3. The results showed the correlations among physical subhealth, risk perception, demographic variables, and control variables.

From Figure 3, it can be seen that physical subhealth was negatively correlated with the living place, marital status, average annual household income, subhealth duration, and physical subhealth risk perception level (*P* < 0.05). The risk perception level was positively correlated with the education level, living place, average annual household income, subhealth duration, number of employees in the work unit, and subhealth proportion in the work unit (*P* < 0.05), and negatively correlated with age (*P* < 0.05). There will be a multicollinearity problem when the correlation coefficient is more than 0.9, and there may be a problem when the correlation coefficient is over 0.8 [24], so 0.6 is the baseline for an acceptable correlation coefficient [25]. In this study, only the correlation coefficient between age and working years and that between age and number of children exceeded 0.6, and both correlation coefficients were 0.66. We conducted a multicollinearity test on all data. The larger the variance inflation factor (VIF), the greater the problem of multicollinearity. More specifically, multicollinearity is not a problem when the tolerance value is greater than 0.10 and the variance inflation factors (VIFs) are less than 10. In our study, the lowest tolerance value was 0.354 and the highest VIF was 2.829. Accordingly, multicollinearity does not appear to be a significant problem in our dataset.

### 3.4. Regression Analysis

The multiple stepwise regression model for physical subhealth and risk perception level on the demographic characteristic variables and control variables is provided in Table 3.

The article "An Empirical Study on Physical Subhealth Risk Perception: A Physical Examination Data of Tertiary Grade-A Hospitals in Anhui Province, China" was published in 2023. Journal: J Environ Public Health.

It can be seen from Table 3 that age, education level, and the subhealth proportion in the work unit had a significant positive influence on the physical health (*P* < 0.05), while the living place, marital status, and subhealth duration significantly and negatively influenced the physical health of the examinees (*P* < 0.05). The living place, average annual household income, number of employees in the work unit, and subhealth proportion in the work unit had a significant positive influence on the level of risk perception (*P* < 0.05), while age had a significant negative influence on the level of risk perception (*P* < 0.05).

The results in Figure 2 partially supported Hypothesis 1: The risk perception level has an impact on physical subhealth.

The results in Figure 3 showed that there is a significant negative correlation between physical health and risk perception level. Therefore, Hypotheses 1 and 2 are partially supported.

Figure 3 and Table 3supported Hypotheses 3 and 4. Some demographic variables and control variables have significant effects on physical subhealth and risk perception.

### 3.5. Moderating Effects among the Study Variables

We used two-way interactions in a moderated multiple regression to explore the moderating effect of demographic variables and control variables on physical subhealth and the risk perception level (Table 4). The results showed that among the abovementioned variables, only the number of children of physical examinees had a significant moderating effect on physical subhealth and risk perception level (*P* < 0.05). The specific moderating efficiencies are shown in Figure 4.

As shown in Figure 4, the risk perception level of physical examinees with more children and higher health level was significantly lower than those with fewer children. The risk perception level was higher in families with fewer children than in families with more children. The poorer the level of physical health, the higher the level of risk perception. Meanwhile, the difference between the two groups of samples was small, the possible reason was that our study only considered the impact of the number of children on the physical health and risk perception level of the physical examinees, and did not consider the age of the children. The family burden of the children of different ages was different. The age of the children in this study may be relatively similar, so the difference between the two samples was small.

## 4. Discussion

The purpose of this study was to explore the relationships between risk perception level, demographic characteristics, and physical subhealth among physical examinees. Furthermore, the roles of demographic variables as moderators in the relationship between risk perception level and physical subhealth were investigated.

The article "An Empirical Study on Physical Subhealth Risk Perception: A Physical Examination Data of Tertiary Grade-A Hospitals in Anhui Province, China" was published in 2023. Journal: J Environ Public Health.

From Figure 3, it can be seen that the physical health status and the risk perception level of the study participants were significantly and negatively correlated. On the one hand, when the risk perception level of the study participants increased above the normal level, they became more worried about their health, which further caused psychological anxiety and tension [26]. Physical subhealth is often an outward manifestation of psychological subhealth. More psychological pressure can lead to the growth of negative emotions [27]. Studies have found that anxiety and depression can reduce the subjective sense of health of the public, increase the degree of physical and mental discomfort of the public [28], and take their physical health into a low-quality state. On the other hand, as physical subhealth deepens, the public's internal anxiety and worry can raise the risk perception level. Based on these results, we put forward the following suggestions. First, decision-makers should pay attention to public mental health and correctly guide public risk perception. For groups with low levels of physical subhealth risk perception, leaders should target and push physical subhealth prevention knowledge through technology software or programs such as WeChat applets and relative health APPs to improve the public's physical subhealth perception level. For groups with high levels of risk perception, information about physical health checkups and health care knowledge should be publicized.

The study results show that age, education level, and subhealth proportion in the work unit all significantly and positively influence physical health, whereas living place, subhealth duration, and marital status negatively influence physical health. One of the possible reasons for the results is that most of the physical examinees in this study are under 45 years of age (83%); fewer are elderly. With the improvement of living standards, contemporary young people are more concerned about their health, so it is understandable that age has a positive effect on physical health in this study. Later, the scope of the study participants could be expanded to increase the data for the elderly group. A second possible reason is that the study participants with higher education level mainly focus on their own and family's quality of life and are more willing to spend money and time to buy health care products or exercise, so they have a relatively better physical health status. So, we encourage the public to attach importance to education. A third possible reason is that the higher the subhealth proportion in the work unit of the study participants, the more risks the study participants perceive, and they will take various measures to improve their health status actively. A fourth possible reason is that people living in second-tier developed cities have a more stressful and faster life and encounter serious environmental pollution, both of which lead to poorer physical health. Therefore, we propose to improve the public living environment to build a livable city. A fifth possible reason is that divorce has become more common in recent years, unhappy marital status (e.g., divorce) and discordant family life indirectly induced physical subhealth conditions due to psychological imbalance, negative emotions, and increased stress [29]; our results are consistent with the studies of Lopez et al. [30]. Based on this, it is recommended that the relevant marriage laws should be improved and the implementation of a divorce cooling-off period should be implemented. We must strengthen psychological guidance and intervention for couples heading toward divorce to reduce the divorce rate. A sixth possible reason is that when the body is in a subhealthy state for a long time without intervention or treatment, the subhealthy condition will gradually worsen and even evolve into a disease. Based on this logic, our result is consistent with Bo-Yang's research to a certain extent [2]. Of course, other possible reasons cannot be ruled out.

The article "An Empirical Study on Physical Subhealth Risk Perception: A Physical Examination Data of Tertiary Grade-A Hospitals in Anhui Province, China" was published in 2023. Journal: J Environ Public Health.

Our analysis of the results shows that the living place, average annual household income, number of employees in the work unit, and subhealth proportion in the work unit significantly and positively influence the risk perception level, and only age negatively influences the risk perception level. One possible reason is that the older the study participants, the greater their life experience and exposure, the better their ability to handle risk, and the lower their physical subhealth risk perception level. Another possible reason is that when people have a more prosperous and developed place of living, a higher household income, and a higher quality of life, then they are more concerned about their health, so they have a higher level of physical subhealth risk perception. Therefore, it is recommended that social resources should be allocated rationally to reduce the gap between the rich and the poor. Yet another possible reason is that more employees in the work unit, higher the subhealth proportion in the work unit indicating a higher number of subhealthy people in the work unit. This will bring psychological panic and anxiety to the study participants. In those conditions, they will worry more about their health status and the level of physical subhealth risk perception will gradually increase. We should focus on the health of work unit employees and regularly organize employees to attend medical checkups.

The article "An Empirical Study on Physical Subhealth Risk Perception: A Physical Examination Data of Tertiary Grade-A Hospitals in Anhui Province, China" was published in 2023. Journal: J Environ Public Health.

Our results show that the number of children of physical examinees had a significant moderating effect on the relationship of physical subhealth and risk perception level. The risk perception level of physical examinees with more children and higher health level was significantly lower than those with fewer children, and the risk perception levels were higher in families with fewer children than in families with more children. A possible reason for the moderation is that examinees with more children and better health spend more time and energy on their children and pay less attention to their own physical health, so it is understandable that the risk perception level of examinees with more children and better health is significantly lower. A second possible reason is that families with fewer children typically have a lower level of economic pressure than families with more children, so they have more energy and financial resources to spend on their own health management. Also, they are often more sensitive to information about their own health status, and once they perceive a change in their health status, they will quickly take countermeasures, so it is not difficult to understand that families with fewer children have a higher level of risk perception. A third possible reason is that when the physical health status of the examinees is poor, their psychological burden will increase, and poor health will also trigger internal panic and anxiety, so the risk perception level of the examinees is correspondingly higher. The number of children in a family is related to China's population policy. China's family planning policy was in force for decades and attracted great attention from the public. The policy has made a remarkable contribution to reduce China's fertility rate, control the total population, and avoid the negative problems caused by overpopulation, but China also needs to face up to the series of problems it brought, such as the accelerated process of population aging and the serious imbalance of the sex ratio at birth [31]. With the continuous development of the economy and society, the progress of medical and health services, and the improvement of people's living standards, China's population is aging [32]. In response to the increasing average age of its population, China has implemented a comprehensive two-child policy to adjust the demographic structure and slow down the aging trend, but the implementation of the policy did not trigger a birth boom among pregnant women of the right age in China. Cha et al. [33] found that after the implementation of the “comprehensive two-child” policy in China, the second-child fertility rate among women of childbearing age did not increase, but remained at a low level, mainly because women of childbearing age in China perceive risks such as high financial pressure, high cost of raising children, unattended children, and impact on work and career development [34, 35]. How to coordinate responses to the aging population and the “comprehensive two-child” policy requires the support and cooperation of relevant government departments. It can also contribute to the development of our public physical health by, for example, promoting the national policy of better prenatal and postnatal care.

The article "An Empirical Study on Physical Subhealth Risk Perception: A Physical Examination Data of Tertiary Grade-A Hospitals in Anhui Province, China" was published in 2023. Journal: J Environ Public Health.

## 5. Conclusion

This study investigated how the risk perception level and demographic characteristics affect physical subhealth among physical examinees. The results showed that the risk perception level and average annual household income were significantly and negatively correlated with the physical subhealth status of the medical examiners. The poorer the level of physical health, the higher the level of risk perception. The level of risk perception had the opposite effect on physical subhealth. Age, education level, living place, marital status, subhealth duration, and subhealth proportion in the work unit were direct influences on physical subhealth. The risk perception level and average annual household income were indirect factors that influenced the physical subhealth status of the examinees. The moderating effect of the number of children on physical subhealth status and risk perception level was significant.

Based on this, we suggest that the overall improvement of public health can be achieved by enhancing public literacy and education level, improving the housing and living environment to build a livable city, strengthening psychological guidance and intervention for couples heading toward divorce to reduce the divorce rate, encouraging the public to attend regular medical check-ups, allocating social resources rationally to avoid unreasonable wage increases, disseminating the national policy on better prenatal and postnatal care, and enhancing the public's awareness of physical health care.

## Figures and Tables

**Figure 1:** Conceptual model.

**Figure 2:** Heatmap of the distribution of physical subhealth rate in different risk perception levels (%).

**Figure 3:** Correlation diagram. *Note*. The larger the shadow circle and the deeper the color, the greater the correlation coefficient (absolute value). The numerical value of the lower left part represents the correlation coefficient between the variables; the upper right shaded circle indicates a significant correlation at the 0.05 level (2-tailed); and the blank parts indicate no significant correlation at the 0.05 level (2-tailed). R1 stands for physical subhealth status; R2 stands for physical subhealth risk perception level; R3 stands for gender; R4 stands for age/years; R5 stands for education level; R6 stands for years of working; R7 stands for living place; R8 stands for marital status; R9 stands for number of children; R10 stands for average annual household income; R11 stands for self-assessment of health; R12 stands for subhealth duration; R13 stands for number of employees in the work unit; and R14 stands for subhealth proportion in the work unit.

The article "An Empirical Study on Physical Subhealth Risk Perception: A Physical Examination Data of Tertiary Grade-A Hospitals in Anhui Province, China" was published in 2023. Journal: J Environ Public Health.

**Figure 4:** Number of children moderation interaction diagram for physical subhealth and risk perception level.

**Table 1:** Demographic variables and encoding.

Variables	Variable name and encoding
Gender	Male = 1 and female = 2
Age (years)	Less than 30 = 1, 30 to 45 = 2, 46 to 60 = 3, and more than 60 = 4
Education level	Primary or below = 1, junior high school = 2, senior high school = 3, junior college = 4, undergraduate = 5, and master's degree and above = 6
Years of working	Less than 5 years = 1, 5 to 10 years = 2, 11 to 20 years = 3, 21 to 30 years = 4, and more than 30 years = 5
Living place	Rural = 1, cities and towns = 2, third-tier city = 3, second-tier city = 4
Marital status	Never married = 1, married = 2, and other (e.g., divorced, widower/widow) = 3
Number of children	Zero children = 1, one child = 2, two children = 3, and three or more children = 4
Average annual household income	Less than 30,000 yuan = 1; 30,000 to 60,000 yuan = 2; 60,000 to 100,000 Yuan = 3; 100,000 to 200,000 yuan = 4; more than 200,000 yuan = 5
Self-assessment of health	More serious than sub-health = −2, sub-health = −1, unclear = 0, and health = 1
Subhealth duration	Less than 3 months = 1, 3 to 6 months = 2, 6 months to 1 year = 3, less than 2 years = 4, more than 3 years = 5
Number of employees in the work unit	Freelance = 1, less than 50 = 2, 50 to 150 = 3, 150 to 500 = 4, more than 500 = 5
Subhealth proportion in the work unit	10% = 1, 30% = 2, 50% = 3, 70% = 4, more than 90% = 5

**Table 2:** Characteristics of demographic variables and control variables of participants.

Variables	Composition ratio (%)	Mean ± SD
*Gender*		1.59 ± 0.49
Male	312 (40.5)	
Female	458 (59.5)	
*Age (years)*		34.5 ± 11.68
<30	384 (49.9)	
30–45	256 (33.2)	
46–60	96 (12.5)	
>60	34 (4.4)	
*Education level*		3.97 ± 1.38
Primary or below	44 (5.7)	
Junior high school	103 (13.4)	
Senior high school	111 (14.4)	
Junior college	146 (19.0)	
Undergraduate	304 (39.5)	
Master's degree and above	62 (8.1)	
*Years of working*		2.17 ± 1.21
<5	306 (39.7)	
5–10	186 (24.2)	
11–20	161 (20.9)	
21–30	74 (9.6)	
>30	43 (5.6)	
*Living place*		3.10 ± 1.19
Rural	117 (15.2)	
Cities and towns	132 (17.1)	
Third-tier city	110 (14.3)	
Second-tier city	411 (53.4)	
*Marital status*		1.69 ± 0.63
Never married	287 (37.3)	
Married	457 (59.4)	
Others	26 (3.4)	
*Number of children*		0.93 ± 0.94
0	315 (40.9)	
1	244 (31.7)	
2	158 (20.5)	
≥3	53 (6.9)	
*Average annual household income (yuan)*		3.09 ± 1.19
<30,000	88 (11.4)	
30,000–60,000	152 (19.7)	
60,000–100,000	227 (29.5)	
100,000–200,000	205 (26.6)	
>200,000	98 (12.7)	
*Self-assessment of health*		−0.64 ± 0.88
Serious than subhealth	67 (8.7)	
Subhealth	499 (64.8)	
Unclear	61 (7.9)	
Health	143 (18.6)	
*Subhealth duration*		3.37 ± 1.43
<3 months	126 (16.4)	
3–6 months	88 (11.4)	
6 months-1 year	161 (20.9)	
<2 years	162 (21.0)	
≥3 years	233 (30.3)	
*Number of employees in the work unit*		2.97 ± 1.46
Freelancer	171 (22.2)	
<50	152 (19.7)	
50–150	141 (18.3)	
150–500	139 (18.1)	
≥500	167 (21.7)	
*Subhealth proportion in the work unit (%)*		2.94 ± 1.16
10	97 (12.6)	
30	174 (22.6)	
50	246 (31.9)	
70	182 (23.6)	
≥90	71 (9.2)	

The article "An Empirical Study on Physical Subhealth Risk Perception: A Physical Examination Data of Tertiary Grade-A Hospitals in Anhui Province, China" was published in 2023. Journal: J Environ Public Health.

**Table 3:** Regression model.

Variables (*N* = 770)	*Step 1*		*Step 2*	
	*β*/Coef	SE	*β*/Coef	SE
*Physical subhealth/health*				
Gender	0.091	0.247		
Age (years)	0.045^*∗*^	0.017	0.028^*∗*^	0.014
Education level	0.245^*∗*^	0.116	0.244^*∗*^	0.106
Years of working	−0.174	0.142		
Living place	−0.425^*∗*^	0.117	−0.433^*∗*^	0.107
Marital status	−0.340	0.241	−0.446^*∗*^	0.226
Number of children	−0.071	0.186		
Average annual household income	−0.081	0.116		
Self-assessment of health	0.069	0.155		
Subhealth duration	−0.324^*∗*^	0.097	−0.354^*∗*^	0.090
Number of employees in the work unit	0.096	0.091		
Subhealth proportion in the work unit	0.235^*∗*^	0.114	0.237^*∗*^	0.111
Adjusted *R*^2^	0.052		0.054	
*F*	4.48		8.338	

*Risk perception level*				
Gender	0.773	0.885		
Age (years)	−0.113	0.062	−0.079^*∗*^	0.038
Education level	−0.061	0.416		
Years of working	0.563	0.509		
Living place	1.586^*∗*^	0.418	1.649^*∗*^	0.405
Marital status	−0.427	0.864		
Number of children	−0.026	0.667		
Average annual household income	1.371^*∗*^	0.416	1.369^*∗*^	0.390
Self-assessment of health	−0.365	0.555		
Subhealth duration	0.143	0.349		
Number of employees in the work unit	0.784^*∗*^	0.326	0.814^*∗*^	0.316
Subhealth proportion in the work unit	0.683	0.408	0.851^*∗*^	0.371
Adjusted *R*^2^	0.091		0.096	
*F*	7.442		17.331	

^*∗*^indicates *P* < 0.05.

**Table 4:** Moderating effects of demographic variables and control variables.

Dependent variables	Independent variables	Moderator variables	Interaction coefficient	Adjusted *R*^2^
Risk perception level	Physical subhealth/health	Gender	0.312	0.0018
		Age (years)	−0.006	0.0003
		Education level	0.041	0.0002
		Years of working	0.167	0.0026
		Living place	−0.156	0.0025
		Marital status	−0.101	0.0003
		Number of children	−0.300^*∗*^	0.0052^*∗*^
		Average annual household income	−0.034	0.0001
		Subhealth duration	−0.018	0.0001
		Number of employees in the work unit	0.024	0.0001
		Subhealth proportion in the work unit	−0.048	0.0002

*Note.* ^*∗*^indicates *P* < 0.05.

The article "An Empirical Study on Physical Subhealth Risk Perception: A Physical Examination Data of Tertiary Grade-A Hospitals in Anhui Province, China" was published in 2023. Journal: J Environ Public Health.

## Data Availability

The data and materials in the current study are available from the corresponding author upon reasonable request.

## References

[1] Qian H. N. (2006). Discussing and analyzing prevention and cure strategy of traditional Chinese medicine according to characteristic of sub-health condition. *China Journal of Traditional Chinese Medicine and Pharmacy*.

[2] Pan B. Y., Chen T., Lei L. M. (2019). Progress of research on massage therapy for sub-health conditions. *TMR Non-Drug Therapy*.

[3] Ren Q., Li W., Ren X., Xu Q., Zhang Z., Xiao Y. (2015). Study on sub-health status and the relationship between it and personal life habits of grade one students in high school in Nanchang City. *Journal of Hygiene Research*.

[4] Jiang X. L., Zhang L. P., Wang P., Du Y., Sun J. (2020). Research progress of doctor-patient risk perception. *American Journal of Applied Psychology*.

[5] Dong Z., Xu T., Li Y., Feng P., Gao X., Zhang X. Review and application of situation awareness key technologies for smart grid.

[6] Huang C., Vaneckova P., Wang X., FitzGerald G., Guo Y., Tong S. (2011). Constraints and barriers to public health adaptation to climate change. *American Journal of Preventive Medicine*.

[7] VanDyke S. D., Shell M. D. (2017). Health beliefs and breast cancer screening in rural appalachia: an evaluation of the health belief model. *The Journal of Rural Health*.

[8] Khorsandi M., Fekrizadeh Z., Roozbahani N. (2017). Investigation of the effect of education based on the health belief model on the adoption of hypertension-controlling behaviors in the elderly. *Clinical Interventions in Aging*.

[9] Bubeck P., Wouter Botzen W. J., Laudan J., Aerts J. C., Thieken A. H. (2018). Insights into flood-coping appraisals of protection motivation theory: empirical evidence from Germany and France. *Risk Analysis*.

[10] Ling M., Kothe E. J., Mullan B. A. (2019). Predicting intention to receive a seasonal influenza vaccination using Protection Motivation Theory. *Social Science & Medicine*.

[11] Wright D. R., Lozano P., Dawsonhahn E., Christakis D. A., Haaland W. L., Basu A. (2016). Parental predictions and perceptions regarding long-term childhood obesity-related health risks. *Academic Pediatrics*.

The article "An Empirical Study on Physical Subhealth Risk Perception: A Physical Examination Data of Tertiary Grade-A Hospitals in Anhui Province, China" was published in 2023. Journal: J Environ Public Health.

[12] Renner B., Gamp M., Schmälzle R., Schupp H. T. (2015). Health risk perception. *International Encyclopedia of the Social & Behavioral Sciences*.

[13] Källberg A. S., Ehrenberg A., Florin J., Ostergren J., Goransson K. E. (2017). Physicians’ and nurses’ perceptions of patient safety risks in the emergency department. *International Emergency Nursing*.

[14] Ban J., Huang L., Chen C., Guo Y., He M. Z., Li T. (2017). Integrating new indicators of predictors that shape the public’s perception of local extreme temperature in China. *Science of the Total Environment*.

[15] Yang B., Qin Q. Z., Han L. l., Lin J., Chen Y. (2018). Spa therapy (balneotherapy) relieves mental stress, sleep disorder, and general health problems in sub-healthy people. *International Journal of Biometeorology*.

[16] Wang B., Yang S., Huang Z., Li D., He J., Wang X. (2018). Data mining-based subhealth analysis of Chinese software programmers in 2017. *Informatics in Medicine Unlocked*.

[17] De Santis J. P., Hauglum S. D., Deleon D. A., Provencio-Vasquez E., Rodriguez A. E. (2016). HIV risk perception, HIV knowledge, and sexual risk behaviors among transgender women in south Florida. *Public Health Nursing*.

[18] Essien E. J., Ogungbade G. O., Ward D., Fernandez-Esquer M., Smith C., Holmes L. (2008). Injecting drug use is associated with HIV risk perception among Mexican Americans in the Rio Grande Valley of South Texas, USA. *Public Health*.

[19] Essien E. J., Ogungbade G. O., Ward D. (2007). Influence of educational status and other variables on human immunodeficiency virus risk perception among military personnel: a large cohort finding. *Military Medicine*.

[20] Adedimeji A. A., Omololu F. O., Odutolu O. (2007). HIV risk perception and constraints to protective behaviour among young slum dwellers in Ibadan, Nigeria. *Journal of Health, Population and Nutrition& Nutrition*.

[21] Sun J. J., Jiang X. L., Gao Y. F. (2022). Subhealth risk perception scale: development and validation of a new measure. *Computational and Mathematical Methods in Medicine*.

[22] China Association of Chinese Medicine (2006). *Clinical Guidelines of Chinese Medicine on Sub-health*.

[23] Zhang Y. H. (2009). The calculation of quartiles in statistics. *China High-Tech Enterprise*.

[24] Sun J. J., Wang P., Du Y. N., Liu J. (2020). Analysising the influence factors of single task pricing based on public packet system: an Empirical Study in China. *Journal of Physics: Conference Series*.

[25] Sun J. J., Sun R., Jiang Y. (2020). The relationship between psychological health and social support: evidence from physicians in China. *PLoS One*.

The article "An Empirical Study on Physical Subhealth Risk Perception: A Physical Examination Data of Tertiary Grade-A Hospitals in Anhui Province, China" was published in 2023. Journal: J Environ Public Health.

[26] Liang L., Guo F., Jiang L. (2019). Prevalence and influencing factors of physical sub-health among young and middle-aged police officers in China. *China Journal of Public Health*.

[27] Tang Y. L., Zhang Q. H., Xiong Y. Q. (2015). Health status of 587 police officers in Jiangmen City and its influencing factors. *South China Journal of Preventive Medicine*.

[28] Acquadro Maran D., Varetto A., Zedda M., Ieraci V. (2015). Occupational stress, anxiety and coping strategies in police officers. *Occupational Medicine*.

[29] Xie J., Luo H. B., Zhu H. (2016). Prevalence and influence factors of sub-health among urban residents in Tianjin. *Chinese Journal of Public Health*.

[30] Lopez J. P., Kos A., Turecki G. (2018). Major depression and its treatment: micro RNAs as peripheral biomarkers of diagnosis and treatment response. *Current Opinion in Psychiatry*.

[31] Dou X. (2020). Research on the problems and countermeasures of implementing the comprehensive two child policy in China. *Economic Research Guide*.

[32] Chu H. J. (2020). Rural endowment under the background of aging: current situation, problems and Countermeasures. *Inner Mongolia Science Technology & Economy*.

[33] Cha L., Zhao B., Liu Y. Y. (2020). Intention of having a second child among Chinese females of childbearing age based on China’s universal two-child policy: a meta-analysis. *Chinese Journal of Evidence-Based Medicine*.

[34] Shen X. H. (2017). *Study on the Fertility Desire and Determinant Factors of Childbearing Age Families under the “Comprehensive Two Child” Policy in China*.

[35] Shang L., Huang H. Y., Kou L. L. (2019). Fertility desire and influencing factors of childbearing age women in five provinces and cities in China. *Chinese Journal of Woman and Child Health Research*.

[36] Jiang X., Zhang L., Gao Y., He C., Tang Z., Sun J. (2021). An empirical study on physical sub-health risk perception: physical examination data of tertiary grade-a hospitals in Anhui province, China. https://assets.researchsquare.com/files/rs-154598/v1/60019c23-1b49-422a-8399-a87b8f88fda8.pdf?c=1631878147.

